# Dexmedetomidine Combined with Low-Dose Norepinephrine Continuous Pumping to Prevent Hypotension after Cesaresan Section: A Randomized Controlled Trial

**DOI:** 10.1155/2023/5324055

**Published:** 2023-02-04

**Authors:** Jin Zhang, Jun Chen, Fan Zhang, Yang Song, Quan-Fang Wang, Shao-Lin Wang

**Affiliations:** ^1^Department of Anaesthesiology, The Second People's Hospital of Wuhu, Wuhu 241000, Anhui, China; ^2^Department of Anaesthesiology, The First Affiliated Hospital of Wannan Medical College, Wuhu 241000, Anhui, China

## Abstract

**Objective:**

The aim of the study is to explore the clinical effect of dexmedetomidine combined with low-dose norepinephrine (NE) continuous pumping in preventing supine hypotension.

**Methods:**

A total of 160 puerperaes who underwent elective cesarean section were selected. The puerperaes were equally divided into *S* group (saline), *D* group (dexmedetomidine), *N* group (norepinephrine), and DN group (dexmedetomidine combined with norepinephrine) by a random number table method. Apgar scores and umbilical cord venous blood gas values were recorded at 1 and 5 minutes.

**Results:**

There were no statistically significant differences in the age, gestational age, body mass index, bleeding volume, fluid supplement volume, Apgar scores of new borns at the 1st and 5th minute, the blood gas values of umbilical cord arterial and venous in the four groups (*P* > 0.05). Compared with the *S* group, the incidence of supine hypotension, the number of NE supplements, the supplementary doses of NE, and the incidence of adverse reactions were significantly reduced in the *D*, *N*, and DN groups after spinal anesthesia (*P* < 0.05). Compared with group *D*, the incidence of supine hypotension, the number of additional NE, additional dose of NE, and the incidence of adverse reactions in the DN group after spinal anesthesia were significantly reduced (*P* < 0.05). Compared with the *N* group, the incidence of supine hypotension, the number of additional NE, the additional dose of NE, and the incidence of adverse reactions in the DN group after spinal anesthesia were significantly reduced (*P* < 0.05).

**Conclusion:**

Dexmedetomidine combined with continuous pumping of low-dose norepinephrine can effectively prevent the occurrence of supine hypotension, reduce the occurrence of other adverse reactions, and have no obvious adverse effects on neonates. *Registration.* Chinese Clinical Trial Registry (https://www.chictr.org.cn/enIndex.aspx; ChiCTR2000040979).

## 1. Introduction

Intraspinal anesthesia has always been the first choice for cesarean section. However, after the full-term parturient is anesthetized in spinal canal, the foil effect of abdominal muscles on the uterus is eliminated. In supine position, the enlarged uterus oppresses the inferior vena cava and abdominal aorta. At the same time, anesthesia can dilate the blood vessels in the plane, resulting in supine hypotension syndrome [1]. Intraoperative hypotension is considered to be the main risk factor for perioperative complications such as myocardial ischemia and myocardial infarction and may increase the incidence of postoperative cerebral infarction and postoperative mortality [2]. Dexmedetomidine, as a highly selective *α* − 2 receptor agonist, is used as an adjuvant in anesthesia, which can improve the safety of anesthesia during cesarean section. It has many advantages for parturients after cesarean section, such as preventing nausea and vomiting, reducing stress reaction, and having no adverse effects on newborns [3–5]. Studies have found that when dexmedetomidine is used in general anesthesia, phenylephrine, norepinephrine, and ephedrine can quickly raise blood pressure and correct hypotension caused by compression of vena cava, increase of peripheral resistance, and increase of vagal tension in prone position during general anesthesia [6]. This article aims to explore the clinical effect of dexmedetomidine combined with low-dose norepinephrine (NE) for continuous pumping to reduce blood pressure after cesarean section, and the safety and effectiveness for parturient and newborn.

## 2. Materials and Methods

### 2.1. General Information

This study selected 160 healthy singleton mothers aged 20–35 who underwent elective cesarean section in Wuhu Second People's Hospital from August, 2019, to August, 2021. Participants with cardiovascular disease, fetal congenital malformations, fetal distress and preterm delivery, and participants who have intraspinal anesthesia contradictions were excluded from this study. According to the method of random number table, the patients were equally divided into *S* group (saline), *D* group (dexmedetomidine), *N* group (norepinephrine), and DN group (dexmedetomidine combined with norepinephrine). There were 40 cases assigned for each group. This study was approved by the Ethical Committee of the second People's Hospital of Wuhu, and all patients and their families signed a written informed consent form before the research. The protocol was prospectively registered with the Chinese Clinical Trial Registry (https://www.chictr.org.cn/enIndex.aspx; ChiCTR2000040979).

### 2.2. Study Protocol and Intervention

After all the eligible parturients entered the operating room, venous passage of the upper limb was established, and the left radial artery catheterization was performed under local anesthesia, and BP, HR, EKG and SpO_2_ were monitored continuously. After the parturient was calm, the operating bed was tilted 15° to the left. Group *D* and group DN were injected with dexmedetomidine at a load dose of 0.5 *μ*g/kg. Group *S* and group *N* were injected with normal saline for 10 min. After loading pump, *D* group and DN group were given dexmedetomidine 0.5 *μ*g/kg/h to continue pumping. With the assistance of the anesthesia nurse, the parturient took the right recumbent position and successfully performed epidural puncture in *L*_3-4_ or *L*_2-3_ intervertebral space, and then, the lumbar puncture needle was placed. After the cerebrospinal fluid (CSF) was discharged and extracted without resistance, 1% ropivacaine 1.3 ml (13 mg) + morphine 0.2 ml (0.2 mg) + cerebrospinal fluid 1 ml was injected into the subarachnoid space with a total of 2.5 ml, and the injection speed was 0.1 ml/s. At the same time, norepinephrine 0.04 *μ*g/(kg·min) was injected intravenously in *N* group and DN group. After subarachnoid injection, the lumbar puncture needle was withdrawn, and an epidural catheter at 4 cm was placed into the cranial end. The parturient was quickly converted to a supine position, and the operating bed was tilted to the left 15°. At the same time, the mask inhaled oxygen (5 L/min).

After intrathecal injection of 10 min, the maternal sensory block level was measured by acupuncture method. If the level did not reach T6, 2% lidocaine 5–10 ml was injected through the epidural catheter and exclude the case; if T6 was reached or exceeded, the operation would be started. BP and HR were recorded every minute from immediately after intrathecal injection to 20 minutes after spinal anesthesia. If the maternal SBP decreased by more than 20% or less than 90 mmHg at a single time, it was defined as hypotension and 5 *μ*g of norepinephrine was added intravenously. It was twice recorded that the maternal SBP increased by more than 20% of the base value, which was defined as hypertension. If the maternal hypertension-related symptoms such as headache or SBP were higher than 160 mmHg, the antihypertensive drug (urapidil) was given as appropriate and the pump dose of norepinephrine was reduced. If the heart rate is less than 50 beats/min, intravenous atropine 0.25 mg was given, repeat it if necessary.

### 2.3. Outcome Measures

The primary outcome was defined as the additional dose of NE and the secondary outcome was defined as other indicators of puerperaes and neonates, including the incidence of maternal hypotension. General condition of parturient: age, gestational age, body mass index, volume of bleeding and fluid replacement; intervention dose of norepinephrine and atropine; incidence of maternal hypotension and adverse reactions (reactive hypertension, chest tightness, nausea, shivering, oxytocin reaction); neonatal 1-minute and 5-minute Apgar score [7] and umbilical cord drive, venous blood gas value. Apgar score: 0–3 is severe asphyxia, 4–7 is mild asphyxia, and 8–10 is no asphyxia.

### 2.4. Statistical Analysis

Statistical analysis was performed using SPSS 25.0 software. All data were tested by *K*-*S* test. Quantitative data with normal distribution were expressed as $\left(\bar{x}\;\pm s\right)$, and *t*-test or ANOVA was used to analyze between groups; count data were expressed as examples or percentage, and  *χ*^2^ test was used. Measurements with skewed distribution were expressed as median [*M* (*Q*)], and comparisons between groups were performed using the rank-sum test. *P* < 0.05 means that the difference is statistically significant. The sample size was calculated by the software PASS version 15.0.5. When comparing the main outcomes (additional dose of NE), the two-sided*t*-square test was performed according to *p*=0.05. According to the pre-experimental results, the additional dose of NE in group *N* was supposed as 1.5 ± 2.5 *μ*g, and that in group DN was 0.5 ± 1 *μ*g. When the sample size of *N* group and DN group is 15 cases for each group, the difference can be found with more than 90% confidence.

## 3. Results

### 3.1. Baseline Information and Indicators

The combination of Apgar score and fetal umbilical artery blood gas analysis is considered to be the criterion for judging the state of newborns [8]. In this study, the 1 min Apgar scores of newborns in the four groups were all more than 8, and the 5 min Apgar scores were all 10. All fetal umbilical artery PH, PaO_2_, PaCO_2_ and other indexes are in the normal range, and the difference is not statistically significant. There was no significant difference in age, gestational week, body mass index, amount of bleeding, volume of fluid replacement, Apgar score at 1 minute and 5 minutes, umbilical cord drive and venous blood gas values among the four groups (*P* > 0.05). It is suggested that dexmedetomidine combined with continuous infusion of low dose norepinephrine has no significant adverse effect on newborns (Tables 1 and 2).

### 3.2. Incidence of Hypotension, Additional NE, and Adverse Events

Compared with group *S*, the incidence of hypotension in supine position, the number of additional NE, the additional dose of NE, and the incidence of adverse reactions in group *D*, group *N*, and group DN were significantly lower than those in group *S* (*P* < 0.05). Compared with group *D*, the incidence of hypotension in the supine position, the number of additional NE, the additional dose of NE and the incidence of adverse reactions in DN group were significantly lower than those in group *D* (*P* < 0.05). Compared with group *N*, the incidence of hypotension in supine position, the number of additional NE, the additional dose of NE, and the incidence of adverse reactions in the DN group was significantly lower than those in group *N* (*P* < 0.05) (Tables 3 and 4, Figure 1).

As shown in Figure 2, the incidence of maternal hypotension in group *S* was 52.5%, while that in group *D* was 30%, which was significantly lower than that in group *S*, and the incidence of hypotension after spinal anesthesia in group DN was significantly lower than that in other groups.

The incidence of adverse reactions in the dexmedetomidine group, noradrenalin group, and dexmedetomidine combined with noradrenalin group was significantly lower than that in the saline group, and the incidence of adverse reactions in dexmedetomidine combined with noradrenalin group was the lowest among all groups (2.5%), with only one case of reactive hypertension (Figure 3).

## 4. Discussion

Cesarean section is an important procedure in modern obstetrics. It is of great significance to relieve the anxiety and tension of parturient and reduce the pain and complications of cesarean section patients during perioperative period. Because of the particularity of cesarean section, in order to avoid adverse effects on the fetus, it is particularly important to choose appropriate anesthesia methods and drugs. A meta-analysis found that dexmedetomidine can significantly reduce postoperative chills, while not increasing the incidence of nausea and vomiting during surgery, and there is no obvious bradycardia, and it can enhance sedation [9]. At the same time, some research results show that it has no adverse effects on maternal circulation, labor process, and fetal umbilical artery blood flow, and the safety of mother and baby is good [10].

Spinal anesthesia is more and more favored by obstetricians because of its quick effect, good muscle relaxation effect, completed block, and little effect on the fetus. However, maternal hypotension after spinal anesthesia is a common problem in clinical anesthesia, and its incidence is as high as 80% without any preventive measures [11]. The use of intrathecal dexmedetomidine during cesarean section can shorten the onset time of spinal anesthesia and enhance the effect of local anesthetic. It has no significant impact on neonates and there were no other adverse events [7]. Although postural regulation and fluid expansion can alleviate hypotension after spinal anesthesia, the incidence of maternal hypotension is still high. Therefore, in addition to postural adjustment and fluid infusion, maintaining a certain peripheral vascular resistance and visceral venous tension is the key factor to prevent the decrease of maternal cardiac output in cesarean section anesthesia. Therefore, there are more and more research studies on the application of vasoactive drugs.

Hasanin et al. [12] found that continuous infusion of 0.05 *μ*g/(kg·min) and 0.075 *μ*g/(kg·min) norepinephrine can significantly reduce the incidence of hypotension after spinal anesthesia. Fu et al. [13] adjusted the speed of 0.08 *μ*g/(kg·min) intravenous infusion of norepinephrine according to body weight to prevent hypotension during combined spinal-epidural anesthesia in cesarean section and considered that it could effectively prevent 90% of maternal hypotension. Two recent studies have compared the antihypertensive effects of norepinephrine and ephedrine in spinal anesthesia-balanced cesarean section. Compared with ephedrine, norepinephrine can maintain maternal blood pressure and uterine artery blood flow, and the incidence of intraoperative hypotension and hypertension is low. The frequency of bradycardia and tachycardia is also low, and the amount of norepinephrine used during anesthesia is less than that of ephedrine. During cesarean section, norepinephrine can replace antihypertensive drugs to maintain maternal blood pressure, with no adverse effects on neonatal prognosis. The author believes that through continuous research on the application of norepinephrine in obstetric anesthesia, it is gradually clear that norepinephrine may be more suitable as an adrenergic drug for the prevention and treatment of hypotension after spinal anesthesia than phenylephrine and ephedrine. Jiang et al. [14] found that combined spinal-epidural anesthesia for cesarean delivery, preoperative 10 min intravenous administration of 0.6 *μ*g/kg DEX can maintain maternal heart rate, blood pressure, and other vital signs stable. Kong et al. [15] the addition of DEX to local anesthetics for cesarean section can also keep the hemodynamic stability of the perinatal parturients maternal maintain hemodynamic stability, reduce the incidence of perioperative maternal transient neurological syndrome and postoperative cognitive dysfunction. At the same time, some studies have suggested that dexmedetomidine can effectively reduce the incidence of supine hypotension syndrome during cesarean section and does not cause neonatal asphyxia [1]. Some studies have shown that general anesthesia prone position lumbar surgery combined with dexmedetomidine timing, phenylephrine, norepinephrine and ephedrine can rapidly increase blood pressure and correct hypotension, but the effective pressor effect of ephedrine lasts longer, and the effective pressor effect is accompanied by an increase in CO [6]. Based on the current study, this study used a combination of dexmedetomidine combined with norepinephrine.

According to the previous findings, continuous infusion of norepinephrine 0.04∼0.10 *μ*g/(kg·min) can significantly reduce the incidence of supine hypotension in parturients undergoing cesarean section after spinal anesthesia. The results of Fu et al. [13] show that intravenous injection of 0.04 *μ*g/(kg·min) norepinephrine can reduce the incidence of supine hypotension after spinal anesthesia to 30%, while pump 0.08 *μ*g/(kg·min) norepinephrine can effectively prevent 90% of maternal hypotension after spinal anesthesia. Considering the possible pressor effect of dexmedetomidine, we selected 0.04 *μ*g/(kg·min) as the pump dose in this study. The results showed that the frequency and dose of additional NE and the incidence of postoperative complications in *N* group and DN group were significantly lower than those in the *S* group.

Lankadeva et al. [16] found that dexmedetomidine can enhance the pressor effect of norepinephrine. The mechanism may be that the inhibitory effect of *α*_2_ receptor agonists on the central nervous system can reduce sympathetic activity and reduce the release of endogenous catecholamines from nerve endings. Due to the decrease of the concentration of endogenous catecholamines, the peripheral blood vessels changed from a previously insensitive state to a sensitive state to catecholamines. At this time, exogenous catecholamines can enhance the contractile effect of blood vessels [17]. The results showed that the incidence of supine hypotension in DN group was significantly lower than that in *N* group, which may be related to the pressor effect of norepinephrine induced by dexmedetomidine. Another explanation may be the biphasic effect of dexmedetomidine on hemodynamics. Although dexmedetomidine is a highly selective *α*_2_-adrenoceptor agonist, it can bind to different *α*_2_-adrenoceptors and *α*_1_-adrenoceptors at a certain plasma concentration. Sedation and antisympathetic action on *α*_2*A*_ receptors can lead to a decrease in blood pressure and heart rate, vasoconstriction on *α*_2*B*_ receptors can lead to an increase in blood pressure, and the activation effect of *α*_1_-adrenoceptors can also cause an increase in blood pressure [18, 19]. In this study, the incidence of maternal hypotension in group *S* was 52.5%, while that in group *D* was 30%, which was significantly lower than that in group *S*. This may be due to the high plasma concentration of dexmedetomidine within a few minutes after spinal anesthesia, and the vasoconstriction caused by *α*_2*B*_ and *α*_1_ receptors on peripheral vascular smooth muscle alleviated the vasodilation effect after spinal anesthesia to some extent. After that, with the rapid removal of the fetus, the pressure of the uterus on the inferior vena cava was relieved. Although the mechanisms of vasoconstriction of dexmedetomidine and norepinephrine are different, they cooperate with each other, so that the incidence of hypotension after spinal anesthesia in DN group is significantly lower than that in other groups. Hypotension after spinal anesthesia is an important factor related to chest tightness, nausea, vomiting and other complications [20, 21]. Although norepinephrine was given timely after hypotension, the incidence of adverse reactions in group *S* was still high. In addition to hypotension, it may also be closely related to the use of oxytocin. It has been found that dexmedetomidine can reduce the incidence of gastrointestinal and cardiovascular adverse reactions induced by oxytocin [22, 23]. Therefore, in this study, although the incidence of hypotension in group *D* was higher than that in group *N*, there was no significant difference in the incidence of other adverse reactions between group *D* and group *N*. The DN group had the lowest incidence of adverse reactions and stable circulation during operation.

## 5. Limitation

Although this study has a certain clinical significance, it has certain limitations, and the follow-up needs to be further confirmed by a large-sample, multicenter randomized controlled trial.

## 6. Conclusion

To sum up, in the healthy women who underwent elective cesarean section, continuous infusion of dexmedetomidine combined with low-dose norepinephrine can effectively maintain the circulatory stability of patients during operation, effectively prevent hypotension in the supine position, and reduce the incidence of other adverse reactions, without adverse effect on newborns. When dexmedetomidine combined with low-dose norepinephrine is continuously pumped, attention should be paid to the pump dose of norepinephrine to avoid the corresponding adverse consequences caused by excessive dose.

## Figures and Tables

**Figure 1:** Comparison of additional NE cases, atropine intervention cases, and incidence of hypotension in the four maternal groups. Group *S*: saline; group *D*: dexmedetomidine; group *N*: norepinephrine; group DN: dexmedetomidine and norepinephrine.

**Figure 2:** Additional NE measurement in four maternal groups. Group *S*: saline; group *D*: dexmedetomidine; group *N*: norepinephrine; group DN: dexmedetomidine and norepinephrine.

**Figure 3:** Comparison of adverse reactions in the four maternal groups. Group *S*: saline; group *D*: dexmedetomidine; group *N*: norepinephrine; group DN: dexmedetomidine and norepinephrine.

**Table 1:** Comparison of maternal age, gestational age, body mass index, blood loss, and fluid infusion.

Group	Age	Gestational age (weeks)	BMI (kg/m^2^)	Blood loss (ml)	Fluid infusion (ml)
*S*	27 ± 7	38.7 ± 1.2	27.6 ± 2.5	219 ± 106	303 ± 98
*D*	26 ± 9	39.1 ± 1.0	27.4 ± 2.8	228 ± 108	312 ± 101
*N*	27 ± 5	38.8 ± 1.5	28.5 ± 2.7	231 ± 110	296 ± 104
DN	28 ± 3	38.9 ± 1.4	28.2 ± 2.9	222 ± 109	307 ± 105

Group *S*: saline; group *D*: dexmedetomidine; group *N*: norepinephrine; group DN: dexmedetomidine and norepinephrine. BMI: body mass index.

**Table 2:** Comparison of umbilical cord drive and venous blood gas values among four groups of fetuses.

Position	Group	PH	PaO_2_ (mmHg)	PaCO_2_ (mmHg)	BE (mmol/L)	Lactate (mmol/L)
UV	*S*	7.34 ± 0.04	24.28 ± 4.71	44.52 ± 4.78	0.82 ± 1.26	1.81 ± 0.05
	*D*	7.33 ± 0.10	24.74 ± 4.60	42.18 ± 5.02	0.91 ± 1.12	1.84 ± 0.03
	*N*	7.35 ± 0.11	24.41 ± 4.41	43.21 ± 4.46	0.90 ± 1.07	1.82 ± 0.04
	DN	7.36 ± 0.12	24.39 ± 4.14	43.36 ± 4.32	0.88 ± 1.05	1.78 ± 0.07

UA	*S*	7.29 ± 0.03	14.16 ± 3.77	56.18 ± 5.02	0.44 ± 1.58	2.24 ± 0.57
	*D*	7.29 ± 0.04	14.27 ± 3.17	56.18 ± 5.02	0.46 ± 1.41	2.26 ± 0.49
	*N*	7.28 ± 0.07	14.87 ± 2.93	58.04 ± 6.14	0.51 ± 1.22	2.27 ± 0.46
	DN	7.28 ± 0.10	14.25 ± 2.28	57.12 ± 5.13	0.48 ± 1.37	2.35 ± 0.31

Group *S*: saline; group *D*: dexmedetomidine; group *N*: norepinephrine; group DN: dexmedetomidine and norepinephrine. UA: umbilical artery; UV: umbilical vein.

**Table 3:** Comparison of the incidence of maternal hypotension, the dose of additional NE, and the number of atropine and NE intervention cases.

Group	Incidence of hypotension (*n*, %)	Additional NE cases	Additional atropine cases	Additional NE dose (*μ*g)
*S*	21 (52.5)	21	0	4.1 ± 4.65
*D*	12 (30)	12^a^	1	2.0 ± 2.95^a^
*N*	8 (22.5)	8^a^	1	1.25 ± 2.47^a^
DN	2 (5)	2^abc^	0	0.25 ± 1.01^abc^

Compared with *S* group, *P*^*a*^ < 0.05; compared with *D* group, *P*^*b*^ < 0.05; compared with *N* group, *P*^*c*^ < 0.05. Group *S*: saline; group *D*: dexmedetomidine; group *N*: norepinephrine; group DN: dexmedetomidine and norepinephrine. NE: norepinephrine.

**Table 4:** Comparison of the number of adverse reactions among the four groups of parturients.

Group	Bosom frowsty (*n*, %)	Nausea (*n*, %)	Reactive hypertension (*n*, %)	Shiver (*n*, %)	Oxytocin reaction (*n*, %)
*S*	10 (25)	8 (20)	2 (5)	8 (20)	9 (22.5)
*D*	3 (7.5)^a^	2 (5)^a^	0 (0)	0 (0)^a^	0 (0)^a^
*N*	1 (2.5)^a^	1 (2.5)^a^	1 (2.5)	0 (0)^a^	0 (0)^a^
DN	0 (0)^a^	0 (0)^a^	1 (2.5)	0 (0)^a^	0 (0)^a^

Compared with group *S*, *P*^*a*^ < 0.05. Group *S*: saline; group *D*: dexmedetomidine; group *N*: norepinephrine; group DN: dexmedetomidine and norepinephrine. NE: norepinephrine.

## Data Availability

The datasets used or analyzed during the current study are available from the corresponding author on reasonable request.
